This article has been retracted.

# Foliar application of seed water extract of *Nigella sativa* improved maize growth in cadmium-contaminated soil

**DOI:** 10.1371/journal.pone.0254602

**Published:** 2021-07-12

**Authors:** Madiha Khadim Hussain, Abida Aziz, Hafiza Mamona Allah Ditta, Muhammad Farooq Azhar, Ahmed M. El-Shehawi, Sajjad Hussain, Noman Mehboob, Mubshar Hussain, Shahid Farooq

**Affiliations:** 1 Department of Botany, The Women University, Multan, Pakistan; 2 Department of Forestry, Bahauddin Zakariya University, Multan, Pakistan; 3 Department of Biotechnology, College of Science, Taif University, Taif, Saudi Arabia; 4 Department of Horticulture, Bahauddin Zakariya University, Multan, Pakistan; 5 Department of Agronomy, Bahauddin Zakariya University, Multan, Pakistan; 6 Department of Plant Protection, Faculty of Agriculture, Harran University, Şanlıurfa, Turkey; Ghazi University, PAKISTAN

## Abstract

Cadmium (Cd) is a widespread heavy metal, which commonly exert negative impacts on agricultural soils and living organisms. Foliar application of seed water extract of black cumin (*Nigella sativa* L.) can mitigate the adverse impacts of Cd-toxicity in plants through its rich antioxidants. This study examined the role of seed water extracts of *N*. *sativa* (NSE) in mitigating the adverse impacts of Cd-toxicity on maize growth. Two maize genotypes (synthetic ‘Neelum’ and hybrid ‘P1543’) were grown under 0, 4, 8 and 12 mg Cd kg^-1^ soil. The NSE was applied at three different concentrations (i.e., 0, 10 and 20%) as foliar spray at 25 and 45 days after sowing. All Cd concentrations had no effect on germination percentage of both genotypes. Increasing Cd concentration linearly decreased root and allometric attributes, gas exchange traits and relative water contents of hybrid genotype. However, gas exchange traits of synthetic genotype remained unaffected by Cd-toxicity. Overall, hybrid genotype showed better tolerance to Cd-toxicity than synthetic genotype with better germination and allometric attributes and less Cd accumulation. Foliar application of NSE lowered negative effects of Cd-toxicity on all studied traits, except relative water contents. In conclusion, foliar application of NSE seemed a viable option to improve maize growth in Cd-contaminated soil.

## Introduction

Soil pollution by toxic metals has become one of serious global environmental concern [1]. Heavy metals are accumulated in agricultural lands as a result of anthropogenic activities, including the use of polluted effluents, industrial wastes, phosphate fertilizers, sewage slurry, herbicides and pesticides [2–4]. Cadmium (Cd) is commonly distributed heavy metal in earth crust and ranked at 7^th^ position among the most toxic 20 metals [5–7]. The use of phosphatic fertilizers is the major cause of Cd contamination in agricultural soils [8]. The Cd concentration <0.5 mg kg^–1^ dry weight is regarded as non-toxic, while this concentration may reach up to 3.0 mg kg^–1^ depending upon soil parent material [9]. The Cd concentrations >5–10 μg Cd g^-1^ leaf dry weight is toxic for numerous plant species [10]; however, hyper-accumulator species have the ability to tolerate 100 μg Cd g^-1^ leaf dry weight [11].

Plants can easily uptake Cd from soil, which poses adverse effects on their morphological, physiological, structural and biochemical attributes [4, 12, 13]. The adverse impacts of Cd-toxicity include destruction of thylakoids [14], hindered development [3, 12, 15, 16], leaf chlorosis [12, 17, 18], changed chloroplast ultrastructure and decreased transpiration and photosynthetic rates [19–21]. Cadmium causes negative impacts on all life forms in the soil and moves into harvested parts of plants; thus, enters the food chain [22, 23]. Vegetables consumptions contributes 70–80% of total Cd intake in humans [24–26], which cause serious health hazards [27]. Grazing or ingesting the Cd-polluted fodder by animals and subsequently consumption of milk and meat products cause Cd exposure in human beings [25]. Therefore, lowering Cd uptake in different crops is mandatory to avoid adverse impacts on humans and animals’ health.

Maize (*Zea mays* L.) is an important crop after wheat and rice in Pakistan. The hiking population growth rate of the country is a significant threat to future food security. Therefore, production of the most important crops must be improved to meet the food demands of rapidly growing population in the country. Cell wall of maize plants has a significant potential for binding and retention of toxic metals due to negative charge [28]. Moreover, maize has the ability to accumulate and tolerate a certain Cd concentration without exhibiting toxicity symptoms [3, 29]. Although maize is regarded as a hyper-accumulator, Cd is harmful at high concentration and negatively affect its growth and development [12, 20, 21, 30].

*Nigella sativa* L., a member of the Ranunculaceae, is known as a miracle herb because of its huge antioxidant potential and use in pharmacology [31, 32]. It is used in natural medications and mentioned in several religious books [33]. *Nigella sativa* is commonly used to ameliorate Cd-toxicity in animals [34–37]. Seeds of *N*. *sativa* contain fixed (>30%) and volatile oil (0.40%-0.45%), comprising of 18.4 to 24% thymoquinone [38]. Thymoquinone (2-isopropyl-5-methyl-1, 4-benzo-quinone) is the main volatile component of the seeds [32, 34, 39], which exhibit antioxidant activities and help to overcome Cd-toxicity in animals.

Heavy metal tolerance of different crops is usually improved by chelation [40, 41], foliar application of various plant extracts [42, 43] and use of plants growth promoting rhizobacteria [44–46]. Several studies have reported the defensive role of *N*. *sativa* against harmful effects of heavy metals in animals; however, its role in alleviating Cd-toxicity in plants has been less explored. In a recent study, Ditta et al. [43] reported positive effects of foliar-applied seed water extract of *N*. *sativa* on maize growth grown in chromium (Cr) contaminated soil. Therefore, it was hypothesized that foliar application of *N*. *sativa* seed extract could also improve maize growth under Cd-toxicity.

The present study was conducted to infer the role of different concentrations of *N*. *sativa* seed water extract in improving the growth of maize genotypes under different Cd concentrations. It was hypothesized that i) maize genotypes will differ in their Cd-tolerance level, ii) increasing Cd concentration will suppress the growth of maize genotypes and iii) application of *N*. *sativa* seed extract will improve the growth of maize genotypes and lower Cd uptake. The results will help to improve maize growth on Cd-contaminated soils and help to lower Cd entry in food chain.

## Materials and methods

### Experimental site

This pot study was conducted in the wire house of Agronomy Department, Bahauddin Zakariya University, Multan, Pakistan during 2019 under natural environmental conditions. Round, free-draining, plastic pots with 8 kg filling capacity were used in the experiment. Soil was collected from nearby agricultural lands with no known Cd-toxicity. For soil analysis, three random samples (0–20 cm depth) were collected. The soil analysis indicated that soil was clay-loam with 8.2 pH, 0.87% soil organic matter content, 1.51 dS m^-1^ EC, 0.031%, available nitrogen (N), 140 mg kg^-1^ available potassium (K), 8.00 mg kg^-1^ available phosphorous (P) with none-detectable Cd.

### Experimental details and treatments

The experiment consisted of three different factors, i.e., two maize genotypes, four Cd concentrations and three concentrations of *N*. *sativa* seed water extract (NSE hereafter). Maize genotypes were synthetic ‘Neelum’ and hybrid ‘P1543’. Seeds of synthetic genotype were procured from the market and hybrid genotype were obtained from Pioneer Seeds Sahiwal, Pakistan. Four different Cd concentrations, i.e., 0, 4, 8 and 12 mg Cd kg^-1^ of soil were included in the experiment. Three concentrations of NSE, i.e., 0, 10 and 20% were tested. Cadmium chloride was used as Cd source and mixed well in the soil before the initiation of the experiment. *Nigella sativa* seeds were boiled for 45 minutes to get NSE. The 10 and 20 g seed powder was boiled in 100 ml of water to prepare 10 and 20% NSE, respectively. The NSE was applied as foliar spray at 25 and 45 days after sowing (DAS) in two equal splits. The plants in 0% NSE were sprayed with distilled water only. Four seeds of both genotypes were sown in each pot. The concentrations of NSE were chosen based on the study of Ditta et al. [43]. All treatments had four replications and two pots were considered as a single replicate. This experiment was laid according to completely randomized block design with factorial arrangement. Maize genotypes were main factor, Cd concentration sub factor and NSE was considered as sub-sub factor.

### Crop husbandry

Nitrogenous and phosphatic fertilizers were applied at the rate of 100 and 75 mg/kg soil. The whole P amount was applied at sowing, whereas N was applied in two splits, first at sowing and second split 25 days after sowing. The plants were irrigated with 2 to 3 days interval keeping in view moisture needs. Four grains of furadan (Carbofuron, FMC product) were applied to control maize borers and shoot fly. The plants were harvested 75 DAS.

### Observation germination and early stand formation

The number of germinating seeds were counted daily basis starting from two DAS following Seedling Evaluation Handbook of Association of Official Seed Analysts (AOSA) [47]. Four plants were sown in each experimental pot. The first appearance date of plant was measured as days to start germination for each treatment level. The time take to complete 50% germination (E_50_) was computed according Coolbear et al. [48].


E50=ti+[N2−ninj−ni](tj−ti)

Where, N = final number of germinated seeds, and n_i_ and n_j_ = number of germinated seeds at two adjacent days when n_i_ < N/2 < n_j_.

The formula described by Ellis and Roberts [49] was used to calculate mean emergence time (MET).


MET=ΣDn/Σn

Where, n = number of germinated seeds per day D, and D = number of days totalled from the start of germination.

The number of germinated seeds at final count were converted to percentage and regarded as final germination percentage.

### Growth-related traits

Chlorophyll index was measured at 75 DAS by SPAD meter (Minolta Chlorophyll Meter SPAD-502DL) from all plants, averaged and presented as SPAD values. Likewise, height of all plants from each pot was measured at 75 DAS. Randomly selected one plant from each experimental pot was pulled up carefully at 75 DAS. The leaves were separated and their area was measured with the help of leaf area meter. Shoot fresh weight of uprooted plant was noted from each pot. After sun drying, the samples were placed in oven to dry at 70°C for 48 hr. The shoot dry weight of each pot was noted.

### Relative water contents and gas exchange traits

Leaf relative water contents (RWC) were recorded at 75 DAS. The young fresh leaf was detached from randomly chosen one plant in each replication and weighed fresh. The leaves were then soaked in deionized water for 24 hours to get them completely turgid and weighed to record turgid weight. The leaves were then dried in an over at 75 ± 5°C until constant weight and weighed to record dry weight. Afterwards RWC were calculated by using below formula:

$$Leaf\;RWC\;(\%)=\frac{FW-DW}{TW-DW}\times 100$$

Where, FW = fresh weight of leaf, DW = dry weight of leaf, TW = turgid weight of leaf

Infrared gas analyser LCi-SD portable photosynthesis system (ADC Bio Scientific Ltd. United Kingdom) was used to measure gas exchange traits such as net photosynthetic rate (A), transpiration rate (E) and stomatal conductance (gs) of a single leaf from each pot during 9:00–10:30 am.

### Acid digestion and cadmium analysis

Cadmium accumulation was determined by using the leaves used for the determination of RWC. By using grinding mill, the dried leaves were grinded to fine powder. After two-step acid digestion method [50], the samples were analysed on Atomic Absorption Spectrometer (iCE9 3000 SERIES) to determine Cd accumulation and presented as mg kg^-1^ of plant biomass.

### Statistical analysis

The recorded data of all attributes were tested for normality by Shapiro-Wilk normality test [51], which showed a normal distribution. Thus, the analysis was performed on original data. Fisher’s analysis of variance (ANOVA) technique was used to determine the significance in the data. Two-way ANOVA was used for determining the significance in seedling germination data (since no NSE was applied at germination stage). Data relating to allometric parameters, gas exchange traits, RWC and Cd accumulation were analysed by three-way ANOVA [52]. The LSD (least significant difference test) at 5% probability was used to separate the means where ANOVA showed significant differences. The ANOVA was computed on SPSS version 21 [53]. The data were graphically expressed by Microsoft Excel program through incorporation of standard errors of means.

## Results

### Seed germination and early stand formation

Days to start germination, mean emergence time and final germination percentage of both maize genotypes were not altered by all Cd concentrations. However, the highest Cd concentration significantly increased time taken for 50% germination in both genotypes compared to control (Table 1).

**Table 1:** Effect of different cadmium concentrations on seed germination and early stand establishment traits of two maize genotypes.

Treatments	Time to start emergence (days)	Mean emergence time (days)	E_50_ (days)	Final emergence percentage (%)
Maize Genotypes (M)				
Synthetic	5.2±0.2 A	6.2±0.5 A	5.1±0.2 A	99.3±0.7
Hybrid	4.9±0.1 B	5.7±0.3 B	4.8±0.2 B	100±0.0
LSD value at 5%	**0.17**	**0.38**	**0.18**	**NS**
Cadmium concentrations (mg Cd kg^-1^ soil)				
0	4.9±0.2 B	6.3±0.6	4.7±0.2 B	100±0.0
4	4.9±0.1 B	5.7±0.4	4.8±0.2 B	98.0±1.4
8	5.2±0.2 A	5.9±0.3	5.1±0.2 A	100±0.0
12	5.1±0.0 AB	5.8±0.1	5.1±0.2 A	100±0.0
LSD value at 5%	**0.24**	**NS**	**0.26**	**NS**
M × Cd	**NS**	**NS**	**NS**	**NS**

Means sharing the same case letter for a parameter within a column did not differ significantly from each other at p>0.05.

E_50_ = Time taken to complete 50% emergence; NS = non-significant.

### Growth-related traits

Maize genotypes, Cd concentrations and foliar application of NSE had significant effect (p<0.05) on allometric traits (chlorophyll content, leaf area, shoot dry weight and plant height) of maize (Table 2). Two-way interaction between maize genotypes and Cd concentrations had significant effect, while all other two-way and three-way interactions had non-significant effect on entire growth traits (Table 2).

**Table 2:** Analysis of variance of different growth and biochemical traits of different maize genotypes (synthetic vs hybrid) treated with various black cumin seed extract concentrations (0, 10 and 20%) under different Cd concentrations (0, 4, 8 and 12 mg kg^-1^).

		Chlorophyll content			Leaf area		
SOV	df	SS	MS	*p* VALUE	SS	MS	*p* VALUE
Maize genotype (M)	1	161.40	161.40	0.0010*	1356016	1356016	0.0000*
Cadmium concentrations (Cd)	3	907.26	302.42	0.0000*	2181782	727261	0.0000*
*Nigella sativa* extract (N)	2	234.86	117.43	0.0005*	36013	18007	0.0015*
M × Cd	3	274.39	91.46	0.0006*	45219	15073	0.0012*
M × N	2	16.94	8.47	0.5251^NS^	35816	17908	0.0016*
Cd × N	6	3.81	0.634	0.9995^NS^	40264	6711	0.021*
M × Cd × N	6	8.73	1.46	0.9947^NS^	110443	2401	0.3290^NS^
		**Shoot dry weight (g)**			**Plant height (cm)**		
Maize genotype (M)	1	14.61	14.61	0.0000*	100.35	100.35	0.0013*
Cadmium concentrations (Cd)	3	233.55	77.85	0.0000*	2654.04	884.68	0.0000*
*Nigella sativa* extract (N)	2	3.92	1.96	0.0138*	477.03	238.51	0.0000*
M × Cd	3	19.15	6.38	0.0000*	146.49	48.83	0.0021*
M × N	2	0.025	0.012	0.9706^NS^	12.03	6.01	0.4994^NS^
Cd × N	6	0.268	0.045	0.9952^NS^	96.75	16.13	0.1029^NS^
M × Cd × N	6	0.062	0.010	0.9999^NS^	18.64	3.11	0.8978^NS^
		**Stomatal conductance**			**Photosynthetic rate**		
Maize genotype (M)	1	0.00180	0.00180	0.0197^NS^	0.3850	0.3850	0.8101^NS^
Cadmium concentrations (Cd)	3	0.00278	0.00093	0.0402^NS^	58.501	19.500	0.0420^NS^
*Nigella sativa* (N)	2	0.00058	0.00020	0.3972^NS^	61.530	30.763	0.0143^NS^
M × Cd	3	0.00058	0.00019	0.6048^NS^	33.310	11.104	0.1834^NS^
M × N	2	0.00321	0.00160	0.0092*	1.957	0.9784	0.8625^NS^
Cd × N	6	0.00624	0.00104	0.0077*	68.449	11.408	0.1352^NS^
M × Cd × N	6	0.00807	0.00134	0.0015*	169.87	28.312	0.0016*
		**Transpiration rate**			**Relative water contents**		
Maize genotype (M)	1	0.4232	0.42320	0.0660^NS^	1458.2	1458.2	0.0000*
Cadmium concentrations (Cd)	3	0.8764	0.29212	0.0755^NS^	18844.3	6281.45	0.0000*
*Nigella sativa* (N)	2	0.0862	0.04310	0.6987^NS^	593.1	296.57	0.0127*
M × Cd	3	0.0711	0.02371	0.8967^NS^	12928.3	4309.45	0.0000*
M × N	2	1.1718	0.59590	0.0117^NS^	1.0	0.49	0.9920^NS^
Cd × N	6	2.0633	0.34388	0.0181^NS^	85.7	14.28	0.9642^NS^
M × Cd × N	6	3.1964	0.53274	0.0012*	49.1	8.18	0.9915^NS^
		**Cadmium accumulation**					
Maize genotype (M)	1	0.0338	0.0338	0.0000*			
Cadmium concentrations (Cd)	3	1.1358	0.3786	0.0000*			
*Nigella sativa* (N)	2	0.0271	0.0136	0.0000*			
M × Cd	3	0.0074	0.0035	0.0065*			
M × N	2	0.0006	0.0003	0.5677^NS^			
Cd × N	6	0.0009	0.0002	0.9384^NS^			
M × Cd × N	6	0.0244	0.0005	0.9762^NS^			

Growth-related traits were suppressed by increasing Cd concentrations; however, NSE mitigated the adverse effects to significant extent. Hybrid genotype had higher chlorophyll contents, leaf area and shoot dry weight as compared to synthetic genotype, while the trend was reverse in terms of plant height, relative water content and Cd accumulation (Table 3). The application of 20% NSE resulted in the highest SPAD value, shoot dry weight, plant height, relative water contents and Cd accumulation as compared to control (Table 3). Chlorophyll content, leaf area, shoot dry weight, plant height and relative water content were higher under lower Cd concentration (control) as compared to higher concentrations (Table 3). Mostly higher Cd concentration negatively affected the growth traits (Table 3).

**Table 3:** Effect of different cadmium concentrations on allometric traits, relative water contents and cadmium accumulation of maize genotypes.

Treatments	Chlorophyll content (SPAD value)	Leaf area (cm^2^)	Shoot dry weight (g)	Plant height (cm)	Relative water content (%)	Cadmium accumulation (mg kg^-1^)
	Maize genotypes					
Synthetic	44.7±2.0 B	1498.8±7.7 B	4.30±0.3 B	43.44±1.4 A	70.71±5.0 A	0.27±0.0 A
Hybrid	47.7±1.6 A	1773.3±31.9 A	5.20±0.3 A	41.08±1.6 B	61.71±3.2 B	0.23±0.0 B
LSD at 5%	**1.72**	**23.24**	**0.31**	**1.39**	**3.73**	**0.01**
	***N*. *sativa* seed water extract (%; w/v)**					
0	43.9±1.7 B	1629.2±24.1 A	4.47±0.3 B	39.00±1.5 C	62.48±4.8 B	0.22±0.0 C
10	46.3±1.4 A	1666.2±22.3 B	4.75±0.2 AB	42.50±1.6 B	66.69±3.8 AB	0.25±0.0 B
20	48.4±2.3 A	1612.8±12.9 B	5.04±0.4 A	45.29±1.5 A	69.47±3.7 A	0.27±0.01A
LSD at 5%	**2.10**	**28.47**	**0.37**	**1.70**	**4.56**	**0.01**
	Cadmium levels (mg Cd kg^-1^ soil)					
0	50.8±1.7 A	1857.6±23.6 A	7.60±0.2 A	49.94±1.8 A	80.73±4.1 A	0.42±0.0 D
4	48.4±2.6 B	1731.6±30.9 B	4.79±0.2 B	45.44±1.3 B	75.89±3.3 A	0.31±0.0 C
8	44.1±1.3 C	1557.3±9.5 C	3.88±0.5 C	39.94±1.8 C	69.12±5.4 B	0.31±0.0 B
12	41.7±1.6 C	1397.8±15.1 D	2.73±0.4 D	33.72±1.1 D	39.12±3.5 C	0.42±0.0 A
LSD value at 5%	**2.42**	**32.87**	**0.43**	**1.96**	**5.27**	**0.02**

Means sharing the same case letter for a parameter within a column did not differ significantly from each other at p>0.05.

### Relative water contents and gas exchange traits

Individual effect of genotypes, Cd concentrations and NSE had significant effect (p<0.05) on relative water contents, while photosynthetic rate, transpiration rate and stomatal conductance was non-significantly altered by genotypes, Cd concentrations and NSE application (Table 2). The interactive effect of genotypes, Cd concentrations and NSE had significant effect (p<0.05) on photosynthetic rate, transpiration rate and stomatal conductance (Table 2).

Synthetic genotype showed higher relative water contents as compared to hybrid genotypes. Foliar application of 20% NSE was the most effective in increasing relative water content as compared to control. However, with respect to Cd concentrations, no Cd-toxicity (control) showed higher relative water content as compared to higher Cd concentrations (Table 3).

The highest values of gas exchange parameters, transpiration rate and stomatal conductance were observed under lower Cd concentrations (Figs 1 and 2). Application of 10% NSE improved photosynthetic rate of synthetic genotype, while applications of 10 and 20% NSE had no effect on transpiration rate and stomatal conductance. Gas exchange parameters of hybrid genotype had varied responses. The highest stomatal conductance of hybrid genotype was recorded under no Cd-toxicity, while higher transpiration rate was recorded under lower Cd concentration. However, the highest photosynthetic rate was recorded under higher Cd concentration (Figs 1 and 2). Furthermore, application of 10% NSE resulted in significant improvement in gas exchange traits of hybrid genotype. Overall, hybrid genotype performed better for all parameters than synthetic genotype.

**Fig 1:** Effect of different concentrations of *Nigella sativa* seed extracts on stomatal conductance (A) and photosynthesis rate (B) ± standard errors on maize genotypes grown under various cadmium concentrations. Means sharing the same case letter for a parameter did not differ significantly from each other at p>0.05. Here, NSE = *N*. *sativa* seed extract; DAS = days after sowing.

**Fig 2:** Effect of different concentrations of *Nigella sativa* seed extracts on transpiration rate ± standard errors on different maize genotypes grown under various cadmium concentrations. Means sharing the same case letter for a parameter did not differ significantly from each other at p>0.05. Here, NSE = *N*. *sativa* seed extract; DAS = days after sowing.

### Cadmium accumulation in shoot

Shoot Cd concentration was significantly affected (p<0.05) by genotype, Cd concentrations and NSE concentrations; however, all two and three-way interactions had non-significant effect on shoot Cd concentration (Table 2). Synthetic genotypes observed higher shoot Cd concentration compared with hybrid. Moreover, applications of NSE did not lower shoot Cd concentration in synthetic maize; however, application of 20% NSE significantly lowered the shoot Cd concentration in hybrid maize (Table 3). The higher Cd concentration resulted higher shoot Cd concentration in both maize types as compared to control (Table 3).

## Discussion

The results indicated that different Cd concentrations did not affect seed germination and early stand establishment traits of both genotypes. The possible reasons for non-significant results are that the seeds did not uptake Cd during the germination phase. Stefani et al. [54] suggested that seeds use their own reserves during germination; therefore, it is not effected by the presence of heavy metals in the soil. Due to the reason, germination was not altered by various Cd concentrations included in the current study. Similar results for maize germination under heavy metal stress have been reported in an earlier study [55]. Inhibition of seedling development under Cd-toxicity is dependent on metal concentration in soil [56, 57]. Seed germination of plant species is altered by various environmental factors [58, 59] and large differences exist in different ecotypes of the same species for seed germination [59, 60].

Growth-related parameters of both genotypes were adversely affected by increasing Cd concentration. The highest negative effects on number of roots and root elongation rate were noted in both genotypes under higher Cd concentration. The findings of the current study are supported by other researchers who reported that Cd caused negative effects on maize roots architecture [61, 62]. Alteration in micronutrient uptake in plants under Cd-toxicity is responsible for decrease in protein activity and inhibition of root development [63]. Plant growth rate and plant height of both genotypes were significantly altered by higher Cd concentrations. Similar results have been reported in numerous earlier studies [3, 16, 64]. Cadmium alters protein activity by disturbing the hydrogen-sulphur bond [65]; thus, plants uptake less nutrients and water from roots which hinder development [66]. The growth and productivity of plants are decreased under heavy metals’ stress due to insufficient antioxidant enzymes scavenging ability [67–69].

Higher Cd concentrations caused significant reduction in relative water contents in both genotypes. Decreased relative water contents under Cd stress has also been reported by Farouk et al. [70]. It has been reported that Cd-toxicity causes physiological drought in most plants by disturbing the water relationship between plants, which is responsible for decreased relative water contents [4]. Chlorophyll contents and gas exchange parameters of synthetic and hybrid genotype showed different responses. In synthetic genotype, only photosynthesis was slightly affected by higher Cd concentration. However, chlorophyll contents, transpiration rate and stomatal conductance were not affected under increased Cd concentration. Photosynthetic rate of hybrid genotype remained unaffected by higher Cd concentration; however, chlorophyll contents, transpiration rate and stomatal conductance were negatively affected. Similar results related to Cd-induced decrease in gas exchange traits have been reported for maize and many other plant species [64, 71, 72]. Wu et al. [73] reported that photosynthetic activity of plants is decreased under Cd-toxicity as it disturbs the opening and closing of stomata and damage metabolic processes. Under Cd-toxicity, alteration in gas exchange parameters of maize genotypes may be because of difference in the hereditary material of the maize plants [74].

Foliar application of NSE ameliorated toxic effects of Cd-toxicity and improved growth-related traits and gas exchange parameters of both maize genotypes. Several previous studies have reported that maize and different plant species improved growth and gas exchange parameters by applying foliar application of several substances under metals stress [42, 43, 72]. However, the capacity of NSE to overcome toxic effects of Cd in crop plants has been less explored. A recent study have reported that NSE improved maize growth and related traits under Cr stress [43].

Foliar application of NSE significantly enhanced growth and gas exchange parameters of maize genotypes under Cd-toxicity. The uptake of Cd by cereal crops caused serious health hazards in humans such as different skin issues, kidney failure, high blood pressure and mental variations etc. [4]. *Nigella sativa* has been extensively used in pharmacology [31, 75] and natural remedies [33, 76]. The seeds of *N*. *sativa* possess strong antioxidant activities to scavenge free radicles due to its bioactive components thymoquinone TQ [77, 78]. *Nigella sativa* has been reported to overcome heavy metals toxicity in several animals [34]. Foliar application of NSE mitigated Cd toxicity, which might be due to TQ. However, effective mechanism of NSE involved to improve Cd tolerance needs to be further studied.

The Cd uptake was increased in both genotypes with increasing Cd concentration. Cadmium accumulation in synthetic genotype was higher than hybrid genotype. Similar results are also reported for maize crop [79, 80]. Difference in Cd uptake of maize genotypes may be because of variation in hereditary material [12, 74, 80]. The accumulated Cd even at low concentration is consider as harmful for human ingestion.

## Conclusion

Germination of both maize genotypes remained unaffected under all Cd concentrations, while increasing Cd concentration significantly decreased growth-related traits, gas exchange attributes and relative water contents in both maize genotypes. Gas exchange traits of both genotypes showed different response under Cd-toxicity. Foliar application of NSE ameliorated the toxic effects of Cd-toxicity to significant extent in both genotypes and lowered Cd accumulation. Hybrid genotype had better performance for all traits than synthetic genotype, indicating that hybrid genotype better tolerated Cd-toxicity. Nonetheless, NSE and other plants extracts must also be investigated for their prospective effect in mitigating Cd-toxicity in maize and other crops. However, differential response of gas exchange traits of maize and effective mechanism of NSE involved to improve Cd-tolerance needs to be further studied.
